The article "Therapeutic landscape in mutational triple negative breast cancer" was published in 2018. Journal: Mol Cancer.

# Therapeutic landscape in mutational triple negative breast cancer

**DOI:** 10.1186/s12943-018-0850-9

**Published:** 2018-07-14

**Authors:** Yaqin Shi, Juan Jin, Wenfei Ji, Xiaoxiang Guan

**Affiliations:** 1 Department of Medical Oncology, Jinling Hospital, Medical School of Nanjing University, Nanjing, 210002 China; 2 Department of Medical Oncology, Jinling Clinical College, Nanjing Medical University, Nanjing, 210002 China; 3 Department of Oncology, The First Affiliated Hospital of Nanjing Medical University, Nanjing, 210029 China

**Keywords:** Somatic, Germline, Mutation, Therapeutic, TNBC

## Abstract

Triple negative breast cancer (TNBC) is a heterogeneous disease with aggressive behavior and poor prognosis. Genomic sequencing has detected a distinctive mutational portrait of both the germline and somatic alterations in TNBC, which is staggeringly different from other breast cancer subtypes. The clinical utility of sequencing germline BRCA1/2 genes has been well established in TNBC. However, for other predisposition genes, studies concerning the risk and penetrance to TNBC are relatively scarce. Very few recurrent mutations, including TP53 and PI3KCA mutations, together with a long tail of individually rare mutations occur in TNBC. These combined effects of genomic alterations drive TNBC progression. Given the complexity and heterogeneity of TNBC, clinical interpretation of the genomic alterations in TNBC may pave a new way for the treatment of TNBC. In this review, we summarized the germline and somatic mutation profiles of TNBC and discussed the current and upcoming therapeutic strategies targeting the mutant proteins or pathways to enable tailored-therapeutics.

## Background

### Genomic progress in triple negative breast cancer

Breast cancer is the most frequent malignancy, and causes the second most common cause of cancer death among female [1]. Triple negative breast cancer (TNBC) represents 15% of all breast cancers, but some studies have suggested that its prevalence varies by race and ethnicity. It was reported as high as 39% in Saudi Arabian women [2], 23% in Hispanic population [3], 19% in Chinese [4]. This subtype is associated with aggressive tumor pathology, and poor clinical prognosis [5]. Due to the lack of well-defined molecular targets, the treatment of TNBC relies in chemotherapy, mainly anthracycline, taxanes based regimen. Disease prognosis is poor in patients accompanied by a tendency to develop drug resistance to standard chemotherapy. Improved approaches to treatment of TNBC are highlighted. Advances in next-generation sequencing (NGS) have revealed the genomic complexity and heterogeneity of TNBC. The recent great step was the cluster analysis that identified 6 molecular subtypes displaying unique molecular expression and ontologies. Six TNBC subtypes were proposed as basal-like 1 (BL1), basal-like 2 (BL2), immune modulatory (IM), mesenchymal (M), mesenchymal stem–like (MSL), and luminal androgen receptor (LAR) [5]. Apart from gene clusters, seminal progress has been achieved in mutational spectrum of TNBC related cancer causing genes. These mutational changes, both germline and somatic alterations, contribute to TNBC specific cancer predisposition and progression [6, 7]. Furthermore, TNBC related mutational spectrum shows staggering heterogeneity, extremely distinctive from other types of breast cancer. How to best exploit the genomic alterations of TNBC for therapeutic options remains an important incompletely answered problem. In this review, we summarized a portrait of germline and somatic mutations in TNBC, and focused on investigational therapeutic strategies targeting potential impact somatic or germline alterations, providing valid evidence of future tailored therapy from mutational aspect in TNBC.

The article "Therapeutic landscape in mutational triple negative breast cancer" was published in 2018. Journal: Mol Cancer.

## Main text

### Germline mutations in triple negative breast Cancer

#### BRCA1/2 mutations in TNBC

Compared with other breast cancer, TNBC cases tend to be younger at diagnosis, African American, and BRCA mutation carriers. Patients with TNBC are more likely to have a positive family history [8]. With respect to mostly 60% of *BRCA1* mutation carries displaying a TNBC phenotype [9], *BRCA1* related cancers are closely correlated with TNBC. In contrast, no such association was observed in *BRCA2* mutation carriers.

Previous reviews describing BRCA mutations in TNBC were incomprehensive, for several recent and large cohorts were not included. This review provides more detailed insight (Table 1). Early onset of TNBC, positive family history, and Ashkenazi Jewish (AJ) population are strong predictors for a higher prevalence of BRCA mutations. Two studies in Ashkenazi populations identified a *BRCA1* mutation rate range from 24 to 30% [10, 11]. Besides, in Mexican population, Villarreal-Garza et al. detected a BRCA mutation in 23% of young Mexican women with triple negative breast cancer [12]. Another large cohort assessed the frequency of mutations in 17 breast cancer susceptibility genes in 1824 unselected TNBCs. This study detected higher *BRCA1* mutation rate in patients diagnosed at age<50 years or with family history [3]. Interestingly, in this research, TNBC patients diagnosed over 60 years old have a low BRCA mutation rate (3.1%) [6]. The association between TNBC and BRCA mutations was mostly limited to young patients (Table 1). This supports the general recommendation of BRCA testing in young TNBC patients [6]. However, by performing a retrospective review of 450 racially diverse TNBC referred for genetic counseling, Greenup et al. detected that among patients who were diagnosed with TNBC older than 50, 22.6% of these had either a BRCA1 mutation (14.9%) or a BRCA2 mutation (7.7%). Among patients diagnosed with TNBC older than 60 (*n* = 38), 13% carried BRCA mutations (Table 2) [13]. Besides, in AJ population, a significant proportion of older TNBC patients (>50 years old at diagnosis) carried mutations in BRCA1 (13.9%) and BRCA2 (11.1%) (Table 2) [11]. These observations of a high mutation rate among older TNBC patients support the revised National Comprehensive Cancer Network (NCCN) guidelines to refer patients for BRCA testing based on phenotype. Moreover, the prevalence of genetic mutations among women with TNBC differs significantly by ethnicity. Further researches are warranted to investigate if risk models could include race/ethnicity in risk calculation for patients with TNBC.

The article "Therapeutic landscape in mutational triple negative breast cancer" was published in 2018. Journal: Mol Cancer.

**Table 1:** BRCA1/2 Mutations in Triple Negative Breast Cancer

Reference	Race/Ethnicity	TNBC cases	Total TNBC		TNBC with family history		Early onset TNBC	
			BRCA1 prevalence	BRCA2 prevalence	BRCA1 prevalence	BRCA2 prevalence	BRCA1 prevalence	BRCA2 prevalence
Foulkes 2003 [10]	AJ^a^	72	23.6% (17/72)	0	_	_	_	_
Atchley 2008 [9]	Caucasian/Hispanic/AA^b^/Asian/AJ	93	34.4% (32/93)	7.5% (7/93)	_	_	_	_
Young 2009 [14]	Caucasian/Hispanic/AA/Asian/AJ	54	_	_	_	_	<40 years 16.7%(9/54)	<40 years 1.9%(1/54)
Gonzalez 2011 [78]	Caucasian/Hispanic/AA	77	14.3% (11/77)	3.9% (3/77)	22.7% (5/22)	0	_	_
Comen 2011 [11]	AJ	64	29.7% (19/64)	9.4% (6/64)	BRCA1/2 prevalence 32.1%(9/28)		<50 years 50%(14/28)	<50 years 7.1%(2/28)
Hartman 2012 [79]	Caucasian/Hispanic/AA/Asian	199	6.5% (13/199)	4.0% (8/199)	10.2% (11/108)	4.6% (5/108)	<50 years 9.3%(8/86)	<50 years 5.8%(5/86)
Greenup 2013 [13]	Caucasian/Hispanic/AA/Asian/AJ	450	23.5% (106/450)	7.1% (32/450)	_	_	<40 years 37.7%(55/146)	<40 years 6.8%(10/146)
Sharma 2014 [80]	Caucasian/AA/AJ	207	11.1% (23/207)	4.3% (9/207)	BRCA1/2 prevalence 21.1%(27/128)		BRCA1/2 prevalence: <50 years 27.6%(21/76)	
Couch 2015 [6]	Caucasian/Hispanic/AA/Asian	1824	8.5% (155/1824)	2.7% (49/1824)	13.4% (72/539)	3.2% (17/539)	<50 years 13.0%(98/754)	<50 years 3.6%(27/754)
Tung 2015 [81]	Caucasian/Hispanic/AA/Asian/AJ	87	12.6% (11/87)	1.1% (1/87)	_	_	_	_
Villarreal 2015 [12]	Mexican	190	22.6% (43/190)	0.5% (1/190)	_	_	BRCA1/2 prevalence: <50 years 23.2%(44/190)	
Wong 2015 [82]	Australian	439	5.9% (26/439)	3.4% (15/439)	8.8% (13/147)	2.7% (4/147)	<40 years 11.9%(7/59)	<40 years 3.4%(2/59)
Wong 2015 [82]	Polish	335	5.4% (18/335)	4.5% (15/335)	_	_	<40 years 36.4%(4/11)	<40 years 0
Gonzalez 2016 [83]	Caucasian/Hispanic/AA/Asian	105	12.4% (13/105)	1.9% (2/105)	22.7% (5/22)	9.1% (2/22)	≤50 years 20.8%(11/53)	≤50 years 1.9%(1/53)
Zhang 2016 [84]	Chinese	990	7.2% (71/990)	2.2% (22/990)	_	_	<50 years 10.6%(53/498)	_
Hahnen 2017 [88]	German	291	14.7% (43/291)	2.4% (7/291)	BRCA1/2 prevalence 28.2%(31/110)		BRCA1/2 prevalence: <40 years 35.4%(23/65)	
Sun 2017 [19]	Chinese	1104	7.4% (82/1104)	3.8% (42/1104)	_	_	_	_
Yang 2017 [85]	Malaysians	88	12.5% (11/88)	9.1% (8/88)	_	_	_	_

Abbreviations: ^a^ Ashkenazi Jewish; ^b^ African American

The article "Therapeutic landscape in mutational triple negative breast cancer" was published in 2018. Journal: Mol Cancer.

**Table 2:** BRCA1/2 Mutations in Older Triple Negative Breast Cancer

Reference	Race/Ethnicity	TNBC cases	Total TNBC		TNBC (>50 years)		TNBC (>60 years)	
			BRCA1 prevalence	BRCA2 prevalence	BRCA1 prevalence	BRCA2 prevalence	BRCA1 prevalence	BRCA2 prevalence
Comen 2011 [11]	AJ^a^	64	29.7% (19/64)	9.4% (6/64)	13.9% (5/36)	11.1% (4/36)	_	_
Hartman 2012 [79]	Caucasian/Hispanic/AA^b^/Asian	199	6.5% (13/199)	4.0% (8/199)	4.4% (5/113)	2.7% (3/113)	_	_
Greenup 2013 [13]	Caucasian/Hispanic/AA/Asian/AJ	450	23.5% (106/450)	7.1% (32/450)	14.9% (25/168)	7.7% (13/168)	5.3% (2/38)	7.9% (3/38)
Sharma 2014 [80]	Caucasian/AA/AJ	207	11.1% (23/207)	4.3% (9/207)	BRCA1/2 prevalence 8.4%(11/131)		BRCA1/2 prevalence 4.9%(3/62)	
Couch 2015 [6]	Caucasian/Hispanic/AA/Asian	1824	8.5% (155/1824)	2.7% (49/1824)	3.3% (17/520)	1.3% (7/520)	1.4% (4/279)	0.7% (2/279)
Wong 2015 [82]	Australian	439	5.9% (26/439)	3.4% (15/439)	2.1% (6/286)	3.5% (10/286)	2.2% (4/182)	2.2% (4/182)
Wong 2015 [82]	Polish	335	5.4% (18/335)	4.5% (15/335)	3.5% (10/286)	4.5% (13/286)	2.1% (3/141)	4.3% (6/141)
Gonzalez 2016 [83]	Caucasian/Hispanic/AA/Asian	105	12.4% (13/105)	1.9% (2/105)	3.8% (2/52)	1.9% (1/52)	_	_
Zhang 2016 [84]	Chinese	990	7.2% (71/990)	2.2% (22/990)	3.7% (18/492)	_	_	_

Abbreviations: ^a^ Ashkenazi Jewish; ^b^ African American

In addition, *BRCA2* mutations frequency did not generally increase in young TNBC. Comen et al. observed a frequency of *BRCA2* carriers (9.4%) in 64 Ashkenazi women with TNBC. When identified in patients diagnosed before 50 years old, a lower frequency (7.1%) of *BRCA2* mutations occurred [11]. Greenup et al. also detected a decreased frequency (6.8%) of *BRCA2* mutations in TNBC diagnosed at age<40 years [13]. In Young’s study, only one *BRCA2* mutation in 54 TNBC patients aged<40 years was identified [14]. An increase of *BRCA2* mutation carriers in TNBC was detected with advancing age, and *BRCA2* carriers tended to develop TNBC in older age.

#### Other predisposition genes associated with TNBC

Genetic attributions of other predisposition genes, excluding BRCA1/2 genes, have been limitedly studied, of which, PALB2 and FANCM were more extensively studied (Table 3). In several populations, mutations in PALB2 and FANCM confer the moderate to high risk for breast cancer. Cybulski et al. detected 35 (34%) of 104 PALB2 carriers were triple-negative, while TNBC only accounted for 14% (1257/8928) of breast cancer (p<0.0001) [15]. In Finland, tumors with the PALB2 1592delT mutation were more likely to be triple negative (54.5%, P<0.0001) compared with familiar (12.2%) or sporadic (9.4%) patients [16]. For FANCM mutations, a pronounced association was detected in TNBC patients. Four cases carried FANCM mutations in 215 patients with a TNBC phenotype (OR, 3.75; 95% CI, 1.00–12.85; *P* = 0.02), as compared with the mutation data from German controls [17]. By focusing on the genotyping data of 204 unselected TNBCs, Kiiski et al. reported that FANCM c.5101C>T particularly was enriched, which suggested that FANCM could confer a significant predisposition for TNBC [18].

The article "Therapeutic landscape in mutational triple negative breast cancer" was published in 2018. Journal: Mol Cancer.

**Table 3:** Mutations of other Predisposition genes except BRCA1/2 in Triple Negative Breast Cancer

Reference	Ethnicity/region	TNBC cases	Genes studied except BRCA1/2	Mutations of other predisposition genes	Number of carriers
Wong 2014 [86]	Australia	347 TNBC	PALB2 (Coding regions, intron/exon boundaries)	8 deleterious mutations	41 cases
Cybulski 2015 [15]	Poland	1257 TNBC	PALB2 (c.509_510delGA; c.172_175delTTGT)	_	35 cases
Heikkinen 2009 [16]	Finland	76 familiar TNBC and 56 sporadic TNBC	FANCM (c.1592delT)	_	12 cases
Kiiski 2014 [18]	Finland	204 TNBC	FANCM (c.5101C > T)	_	12 cases
Neidhardt 2017 [17]	Germany	215 non-BRCA mutated, familiar TNBC	FANCM (Coding region)	8 deleterious mutations	4 cases
Ollier 2015 [87]	France	50 non-BRCA mutated, familiar TNBC	36 DNA repair related genes (Coding regions, intron/exon boundaries)	7 deleterious mutation in RAD51D; MRE11A; CHEK2; MLH1; MSH6; PALB2	7 cases
Tung 2015 [81]	Caucasian/Hispanic/AJ/AA/Asian	87 TNBC	23 cancer susceptibility genes (Coding regions, intron/exon boundaries)	3 deleterious mutations in BR1P1; RAD51D; NBN	3 cases
Sun 2017 [19]	China	1104 TNBC	44 cancer susceptibility genes (Coding regions, intron/exon boundaries)	53 deleterious mutations mainly in PALB2, TP53, RAD51D and ATM	53 cases
Couch 2015 [6]	Caucasian/Hispanic/AA/Asian	1824 TNBC	15 other breast cancer susceptibility genes (Coding regions, intron/exon boundaries)	67 deleterious mutations mainly in PALB2, BARD1, BR1P1, RAD51C, RAD51D, RAD50, and XRCC2	67 cases

Apart from studies specially investigating the role of PALB2 and FANCM in TNBC, multiple gene panels including DNA repair related genes or cancer susceptibility genes, were applied to investigate TNBC associated germline mutations. Sun et al. detected the frequency of other breast cancer susceptibility genes (BOCG) mutations (3.8%) in a large series of 1104 TNBC cases [19]. TNBC had the highest prevalence of other BOCG mutations among all breast cancers, in which PALB2, TP53, RAD51D, and ATM were defined as most frequently mutated genes. Besides, Couch et al. reported higher mutation rates (3.7%) of other BOCG mutations in 1824 unselected TNBC patients. Genes participating in DNA repair pathway, mainly PALB2, BARD1, BRIP1, RAD51C, RAD51D, RAD50, and XRCC2, accounted for the highest proportion [6]. These data supported that TNBC mostly was enriched for germline mutations in other predisposition genes among all molecular groups of breast cancer, implying high genome instability and heterogeneity of TNBC.

The article "Therapeutic landscape in mutational triple negative breast cancer" was published in 2018. Journal: Mol Cancer.

Conclusively, more deleterious mutations in multiple genes, including *BRCA1*, *BRCA2* and other predisposition genes are associated with TNBC. The roles and clinical utility of *BRCA* genes have been widely established in clinic. *BRCA1/2* mutation carriers might consider bilateral mastectomy and oophorectomy to lower *BRCA* associated risk. However for other genes, studies concerning the risk and penetrance to TNBC are relatively scarce. There are no available clinical management guidelines for mutations in other predisposition genes except *BRCA1/2*, which urges future research to estimate better cancer risk and establish management guidelines for these mutations.

### Somatic mutations in triple negative breast cancer

#### Distinctive distribution of somatic mutations in TNBC

Advances in NGS have uncovered genomic complexity of breast cancer. The frequency of somatic mutations among breast cancer groups also differs [20]. From data of The Cancer Genome Atlas (TCGA), in luminal A breast cancer, *PIK3CA* was the most frequently mutated genes (45%), followed by mutations in *GATA3* (14%), and mutations in *MAP3K1* (13%), *TP53* (12%). Luminal B cancers mainly have the mutation of *PIK3CA*, *GATA3*, and *TP53*, with the frequency of 29, 15, and 29% respectively. However, TNBC shows a different mutation landscape, with highest frequency of *TP53* mutations, up to 80%, and lowest frequency of *PIK3CA* mutations, which only accounts for 9% [21]. Besides, the loss of tumor suppressor BRCA1, PTEN, and amplification of *MYC* oncogene, present commonly in TNBC [22]. Concurrent *RB1* and *TP53* alterations appear in almost 40% of basal-like breast cancers [23]. Overexpression of *MYC* has been noted with its amplification of 26% in triple negative group.

Recent comprehensive genomic sequencing has suggested a distinctive mutational spectrum across TNBC subtypes [20, 24]. Basal subtype TNBC exhibits more variations than non-basal. *TP53* is more frequently mutated in basal-like TNBC, with nonsense and frameshift mutations enriched. However, mutations in the PI3K pathway tend to appear in non-basal TNBC. Alterations in PI3K signaling in TNBC mainly include mutations in *PIK3CA*, the loss of PTEN and INPP4B [25]. These remind adequate selection of TNBC patients with PI3K pathway activation to PI3K pathway targeted therapy. Except *PIK3CA*, and *TP53*, the majority of other significantly mutated genes in non-TNBC, rarely occur in basal-like TNBC [26]. Apocrine TNBC, a subtype with increased androgen receptor expression, harbors a significantly higher rate of PI3K pathway mutations and *NF1* mutations [27]. However, fewer cases display *TP53* mutations (25%) and *MYC* gains (0%) [27]. Conclusively, these data observed that TNBC displayed a distinctive landscape of somatic genetic alterations among different molecular subtypes. Given these acquired investigations, more researches are needed to detailedly dissect the genetic alterations of specific subtypes in triple negative breast cancer.

The article "Therapeutic landscape in mutational triple negative breast cancer" was published in 2018. Journal: Mol Cancer.

#### Efforts aiming to identify driver mutations in TNBC

Although the genome profiling analysis has provided more comprehensive tools to identify the molecular differences or similarities in breast cancer [28, 29], it speaks little to driver mutations that lead to breast cancer evolution [21, 22]. The continuing advance of NGS has made it possible to systematically identify driving events, which will undoubtedly lead to novel therapeutic targets in TNBC.

Herculean efforts described repertoire of potential driver mutations and mutational processes in breast cancer, and uncovered that novel driver mutations existed in rare groups of patients, making it difficult for their identification, and throwing out challenges to drug discovery and clinical application [30]. In triple negative groups, Shah and colleges investigated the complete mutational and clonal spectrum in 104 early TNBCs [24]. The early TNBC displayed a diverse mutational or clonal landscape, with some exhibiting only a few somatic events and limited pathways, whereas others exhibited hundreds of mutations and involved pathways. Moreover, they revealed that within TNBC, basal subtype tended to exhibit more clonal frequency compared with the non-basal. This study also emphasized driver mutations, including *TP53*, *PIK3CA*/*PTEN*, appeared higher clonal frequency [24]. Banerji and colleagues sequenced to identify recurrent somatic mutations in breast cancer, including *PIK3CA*, *TP53*, *AKT1*, *GATA3*, *MAP3K1*, *CBFB*, and *RUNX1* [31]. In TNBC, a recurrent *MAGI3-AKT3* fusion was identified to activate AKT kinase, suggesting the utilization of AKT small-molecule inhibitors in fusion-positive TNBC patients [31]. Furthermore, there was evidence that novel recurrent structural variations within the enhancer region of *TGFR*, a gene encoding the high affinity ligand for epidermal growth factor receptor (EGFR), occurred in TNBC [32]. Combining with the findings that ectopic expression of *TGFA* promoted cell growth on MCF10A cells, we might consider *TGFA* as a therapeutic target [33]. Anti-EGFR agents as a clinically important implication for TNBC patients should be of particular interest to researchers.

The article "Therapeutic landscape in mutational triple negative breast cancer" was published in 2018. Journal: Mol Cancer.

Conclusively, evidence exhibited tremendous diversity of mutational processes and clonal populations in breast cancer [34]. Researches were also conducted in triple negative group [24]. Integrating these researches enables to subdivide breast cancer and uncover a set of likely driver genes. Despite progress in understanding these driver events, it is still extremely difficult to apply the investigations to clinical use. The immediate significance of these data in clinical application is unknown. More efforts should be conducted upon the functional analysis and clinical identification of these mutations [35].

### Therapeutic strategies from mutational spectrum of TNBC

TNBC remains a breast cancer type with limited options for treatment and a median survival of 19 months [36]. However, a number of therapeutic strategies based on the identification of a few dozen to a few hundred potentially functional impact somatic and germline variants are currently undergoing intensive research [37]. Despite that TNBC is known not to harbor a high frequency of driver mutations, performing a tailored selection of patients with feature of targetable mutant proteins or pathways to individual therapeutic regimens may lead to comparative success in treatment of this heterogeneous disease.

In addition, in the May 2018 issue of *Cell*, Kim et al. showed a herculean effort of single-cell DNA and RNA sequencing in addition to bulk exome sequencing to investigate the genomic and phenotypic evolution of tumor cells in 20 TNBC patients in response to neoadjuvant chemotherapy (NAC), which revealed two distinct groups of clones: clonal extinction and clonal persistence [38]. In the clonal persistence group, patients had residual mutations after treatment. However, in the clonal extinction patients, there were no detectable mutations. Chemotherapy eliminated the tumor cells, leaving only normal diploid cells. Further detailed analysis identified a model of chemoresistance in which both adaptive and acquired evolution cooperated to establish the resistant tumor clones [38]. This study represents a future direction of identifying patients with the chemoresistant-related genomic and phenotypic alterations that could seed metastasis and confer therapeutic resistance, which could contribute to enable better tailored-therapeutics based on genomic profile of TNBC.

The article "Therapeutic landscape in mutational triple negative breast cancer" was published in 2018. Journal: Mol Cancer.

#### Targeting DNA damaging repair pathways

“Omics” based studies have identified a subgroup of TNBC with a deficiency of DNA repair, mainly attributed to mutations or methylation of BRCA1/2, and somatic or germline mutations of other genes involved in DNA damage repair [6, 20, 24]. There is renewed interest of platinum-based chemotherapy in TNBC after preclinical data supporting high benefit of inter-strand cross-linking agents, such as platinum, in BRCA-related subtype. More recently, two large phase 2 randomized trials have provided solid evidence to apply platinum in the adjuvant setting of TNBC: the Geparsixto (NCT01426880) and CALGB40603 (NCT00861705) trials [39, 40]. The Geparsixto trial, in its TNBC subset, 53.2% of 158 patients achieved a pathologic complete response (pCR) with carboplatin, comparatively 36.9% in 136 TNBCs without carboplatin. CALGB40603 reported that the addition of carboplatin with/without bevacizumab to NACT regimen increased pCR rates in 443 TNBC patients. These two studies published the data of disease-free survival (DFS), event-free survival (EFS) and overall survival (OS) recently. In GeparSixto, the addition of carboplatin led to an increase of 3-year DFS by approximately 10%. However, in CALGB40603 trial, no benefit of EFS and OS was observed despite an increased pCR rate [41, 42]. Another TNT trial provided no evidence of unselected advanced TNBC patients more likely to respond to first-line carboplatin than docetaxel, whereas in patients with *BRCA1/2* mutations, carboplatin was superior to docetaxel [43]. These findings suggest earlier tailored therapy for *BRCA*-mutated TNBC in both metastatic and non-metastatic settings.

A proof-of-concept study for poly (adenosine diphosphate-ribose) polymerase (PARP) inhibitors in patients with *BRCA1* or *BRCA2* mutations and advanced breast cancer provided an impressive objective response rate (ORR) of 44% when administrated with olaparib, the mostly investigated PARP inhibitor [44]. Further confirmation in the superiority of PARP inhibitor was conducted in EORTC 1307/BIG 5–13 (BRAVO; NCT01905592; niraparib), EMBRACA (NCT01945775; talazoparib), and OlympiAD (NCT02000622; olaparib). The recent OlympiAD trial detected a longer PFS of 7.0 months in olaparib group than 4.2 months (HR = 0.58, 95%CI: 0.43–0.80,p<0.001) in the standard-therapy group in *BRCA* mutated and HER-negative metastatic breast cancer [45]. The response rate was obviously higher in olaparib group (59.9%) than standard-therapy group (28.8%). With respect to most *BRCA1/2* carriers attributing to TNBC, olaparib could provide a significant benefit among TNBC patients deficient in DNA damage repair. Moreover, we support a promising future of the combination use of PARP inhibitors and platinum in *BRCA* mutated TNBC based on the positive finding from I-SPY2 trial of veliparib-carboplatin [46]. Except *BRCA1/2*, most germline mutations associated with TNBC are mainly distributed in DNA damage repair pathway. As described above, these genes include *PALB2*, *FANCM*, *RAD51D*, *CHEK2*, and others. Therapy design for these mutated genes is scarce. We support the utility of DNA cross-linking agents in combination with targeted agents to improve curative effect for this particular group.

The article "Therapeutic landscape in mutational triple negative breast cancer" was published in 2018. Journal: Mol Cancer.

#### Overriding TP53 mutations related chemotherapy insensitivity

TNBC frequently harbors somatic mutations in *TP53*, a pivotal factor involved in arresting cells in execution of DNA damage response. Loss of p53 conferred chemotherapy resistance in cancer [47], which is partly responsible for the poor prognosis of TNBC. The insensitivity could be reversed by the override of cell cycle checkpoints, which includes direct inhibition of DNA damage significant kinases ATM, ATR, CHK1/2 or wee1 [48, 49]. The inhibition of ChK1 causes abrogation of the G2/M checkpoint in p53-deficient cells with a dysfunctional G1/S checkpoint, thus sensitizing tumors to cytotoxic agents. Since TNBC is extremely associated with *TP53* mutation, in HIM TNBC xenograft model, Cynthia and colleges proved that combination therapy with irinotecan and Chk1 inhibitor (either UCN-01 or AZD7762) induced checkpoint bypass and apoptosis in *TP53* mutated tumors [50]. Multiple clinical trials investigating the efficacy of DNA damaging agents combined with Chk1 inhibitor in solid tumor showed promise for TNBC [51, 52]. Despite an unimpressive clinical activity in a phase 2 study of UCN-01 in 25 metastatic TNBC patients, the failure could be attributed to the low pharmacokinetic property of UCN-01 [53]. Another phase 2 trial (NCT02203513) of LY2606368, another Chk1 inhibitor, in patients with germline *BRCA* mutations or TNBC, is currently being conducted. We are looking forward to future results.

#### Inhibition of PI3K-AKT-mTOR pathway

The homeostasis of PI3K-AKT signaling pathway is mostly broken by the mutations or amplifications of genes encoding the PI3K catalytic subunits (*PIK3CA, PIK3CB*), PI3K regulatory subunit (*PIK3R1*), PI3K effectors (*AKT1, AKT2, PDK1*), AKT-independent mTOR pathway activator (*STK11*) and the loss of PTEN and INPP4B [25]. However, in TNBC, with the relatively low frequency of *PIK3CA* mutations, the loss of PTEN and INPP4B are higher altered in this group compared with other subtypes [54]. Both the M and LAR subtype frequently harbors frequent aberrations in PI3K pathway. Cell lines in these two subtypes preferentially responded to the dual PI3K/mTOR inhibitor NVP-BEZ235 [5]. Furthermore, PI3K signaling pathway can stabilize DNA double-strand breaks and preserve DNA homologous repair state [55]. In BRCA-proficient TNBC model, PI3K inhibition was proven to induce DNA damage, downregulate BRCA1/2, and subsequently sensitized cells to PARP inhibitors. In effect, this inhibition created a BRCA-deficient state [56]. Despite lower frequency of *PIK3CA* mutations in TNBC, targeting TNBC with the activation of PI3K-AKT-mTOR pathway provides clinical benefit in this subgroup. Current clinical trials (NCT01629615; NCT01790932) of the pan-PI3K inhibitor BKM120 have been conducted to investigate the benefit of single agent BKM120 in metastatic TNBC. A further setting in which the pan-PI3K inhibitor BKM120 or PI3Kα selective inhibitor BYL-719 is combined with PARP inhibitor has been carried out to evaluate in recurrent TNBC (NCT01623349).

The article "Therapeutic landscape in mutational triple negative breast cancer" was published in 2018. Journal: Mol Cancer.

Blocking agents aiming at the mTOR kinase are the most studied drugs. Everolimus, as a rapamycin analog, was pronounced in patients with activated PI3K pathway [57, 58]. Preclinical studies in TNBC have validated that the anti-mTOR agents could sensitize basal like breast cancers to cytotoxic drugs or PARP inhibitors [59]. In a BRCA-competent TNBC model, GDC-0980, a dual inhibitor of PI3K and mTOR sensitized the utility of ABT-888 and carboplatin, implying PI3K-AKT-mTOR pathway being involved in DNA damage repair (DDR) mediated antitumor activity of PARP inhibitor in TNBC [60]. Clinical trials of everolimus have been carried out in TNBC patients with some results brought out. A phase 2 trial in primary TNBC randomized 50 patients to receive T-FEC (paclitaxel, 5-fluorouracil, epirubicin, and cyclophosphamide) with/without everolimus. Twelve-week response rate were obtained for the everolimus arm and non-everolimus arm (48% versus 30%) [61]. In another phase 1 trial of mTOR inhibition combined with doxorubicin and bevacizumab for 52 metaplastic TNBC patients, Notable objective response was limited to patients with PI3K pathway alterations. Alterations of PI3K pathway were associated with objective response [62]. Together, these promising data warrants further selection of TNBC patients with activated PI3K-AKT-mTOR pathway to receive PI3K inhibitors or mTOR inhibitors.

The article "Therapeutic landscape in mutational triple negative breast cancer" was published in 2018. Journal: Mol Cancer.

#### Targeting EGFR pathway

Clinical trials of EGFR-targeted TKIs targeting *EGFR* amplification in TNBC generally failed to yield promising results with the use of TKI monotherapy or in combination with chemotherapy [63, 64]. However, in lung cancer, the success of EGFR-targeted TKIs was achieved due to the antitumor activity in tumors harboring activating mutations in tyrosine kinase domain. We suspect the efficacy of TKIs in TNBC mainly attributed to patients with EGFR activating mutations. Most studies detected a rare frequency of activating EGFR mutations in TNBC, whereas we found a discrepant and controversial incidence of EGFR mutations in TNBC between East Asians and Caucasians. In European and Australian research, no or low activating EGFR mutations were identified [65, 66]. In contrast, two studies from Asia detected high EGFR mutation frequencies of 11.4% (8/70) and 7.7% (1/13) in TNBC or basal like cancers separately [67, 68], whereas other studies found no evidence of EGFR gene activating mutations in Japanese and Chinese cohorts [69, 70]. It is still controversial if the same discrepancy of EGFR mutations among ethnicities, which has been reported in lung cancer, exits in TNBC. More efforts will be required to investigate if a portion of TNBC patients may respond to TKI agents.

#### Therapeutics for other potential mutations

Rb is frequently lost in TNBC due to inactivating mutations of *RB1* or loss of heterozygosity (LOH) [71]. Rb deletion cooperating with mutations in *TP53*, lead to aggressive, epithelial-to-mesenchymal transition (EMT)-type tumors. Rb loss is not directly druggable and restoration of Rb function following mutation or deficiency is not feasible. However, targeting its downstream could be actionable. In preclinical model, Rb deficiency coordinated cell cycle progression, and simultaneously increased mitochondrial protein translation (MPT), which sensitized tumor cells to the MPT antagonist tigcycline (TIG). This points to a vulnerability of RB1-deficient TNBC to be treated with TIG, or other MPT inhibitors, which needs to be investigated in clinical settings of RB1-deficient TNBC [23]. Furthermore, given that Rb-deficient cells express high levels of pro-apoptotic factors, therapeutic induction of E2F1, or other pro-apoptotic factors may specially kill Rb-deficient cells [72]. Additionally, therapeutic strategies aiming at the signaling processes associated with Rb deficiency, including hypoxia, glycolysis and EMT process, may be promising approaches to the treatment of Rb deficient cells.

Activating mutations of the genes involved in RAF-MEK1/2-ERK1/2 signaling are quite infrequent in TNBC, and only occur in<5% TNBC cases [26, 73]. Ras/MAPK activity can be aberrantly stimulated via the overexpression of RTKs or copy number alterations of *KRAS* and *BRAF*. Also, loss of DUSP4 or somatic alterations of *NF1* in TNBC can contribute to the activation of RAF/MEK/ERK pathway [74, 75]. Preclinical studies have demonstrated that basal type breast cancer cells have an activated RAS-like transcriptional program and are significantly more sensitive to MEK inhibitors compared with luminal and HER-2 amplified lines. Basal-like cells are more likely to harbor mutations in *BRAF*, *HRAS*, or *KRAS* [76]. Treatment with MEK inhibitor caused the up-regulation of PI3k signaling, and dual inhibition of both pathways could achieve better anti-tumor effects both in vitro and in vivo [77]. These studies provide a rational hypothesis of patient selection in clinical trials seeking to evaluate the clinical effect of MEK and PI3K inhibitors in TNBC.

The article "Therapeutic landscape in mutational triple negative breast cancer" was published in 2018. Journal: Mol Cancer.

## Conclusions

Germline or somatic mutations could shed light on the treatment of TNBC. TNBC deficient in DNA damage repair due to germline mutations could preferentially respond to DNA cross-linking agents, or PARP inhibitors. Tumors with altered PI3K pathway are more likely sensitive to PI3K/mTOR inhibitors. TNBC with TP53 mutations could restore its sensitivity to chemotherapy by targeting cell cycle checkpoints (Fig. 1). Given the limited therapeutic effect of one pathway inhibition in targeted therapy, multi-gene mutational profiles in single patient may increase the opportunity for application of combining two or more targeted agents with the tolerated toxicities [78–88].

**Fig. 1:** TNBC: The current and upcoming therapeutic strategies targeting the mutant proteins or pathways to enable tailored-therapeutics. Therapeutics target at genetic alterations include defects in DNA damage repair, TP53 mutations, activation of PI3K pathway, EGFR amplification/mutations, activation of RAF-MEK signaling, and Rb loss. These genetic alterations were summarized in the white boxes of the diagram. Potential therapeutic strategies were depicted in red boxes

## Abbreviations

AJ: Ashkenazi Jewish
BL1: Basal-like 1
BL2: Basal-like 2
BOCG: Other breast cancer susceptibility genes
DFS: Disease-free survival
EFS: Event-free survival
EGFR: Epidermal growth factor receptor
IM: Immune modulatory
LAR: Luminal androgen receptor
LOH: Loss of heterozygosity
M: Mesenchymal
MPT: Mitochondrial protein translation
MSL: Mesenchymal stem–like
NGS: Next-generation sequencing
ORR: Objective response rate
OS: Overall survival
PARP: Poly (adenosine diphosphate-ribose) polymerase
TCGA: The Cancer Genome Atlas
TNBC: Triple negative breast cancer

## References

[1] Siegel RL, Miller KD, Jemal A (2017). Cancer statistics, 2017. CA Cancer J Clin.

The article "Therapeutic landscape in mutational triple negative breast cancer" was published in 2018. Journal: Mol Cancer.

[2] Al-Tamimi DM, Bernard PS, Shawarby MA, Al-Amri AM, Hadi MA (2009). Distribution of molecular breast cancer subtypes in middle eastern-saudi arabian women: a pilot study. Ultrastruct Pathol.

[3] Lara-Medina F, Perez-Sanchez V, Saavedra-Perez D, Blake-Cerda M, Arce C, Motola-Kuba D, Villarreal-Garza C, Gonzalez-Angulo AM, Bargallo E, Aguilar JL (2011). Triple-negative breast cancer in Hispanic patients: high prevalence, poor prognosis, and association with menopausal status, body mass index, and parity. Cancer.

[4] Lin Y, Yin W, Yan T, Zhou L, Di G, Wu J, Shen Z, Shao Z, Lu J (2009). Site-specific relapse pattern of the triple negative tumors in Chinese breast cancer patients. BMC Cancer.

[5] Lehmann BD, Bauer JA, Chen X, Sanders ME, Chakravarthy AB, Shyr Y, Pietenpol JA (2011). Identification of human triple-negative breast cancer subtypes and preclinical models for selection of targeted therapies. J Clin Invest.

[6] Couch FJ, Hart SN, Sharma P, Toland AE, Wang X, Miron P, Olson JE, Godwin AK, Pankratz VS, Olswold C (2015). Inherited mutations in 17 breast cancer susceptibility genes among a large triple-negative breast cancer cohort unselected for family history of breast cancer. J Clin Oncol.

[7] Dillon JL, Mockus SM, Ananda G, Spotlow V, Wells WA, Tsongalis GJ, Marotti JD (2016). Somatic gene mutation analysis of triple negative breast cancers. Breast.

[8] Kwan ML, Kushi LH, Weltzien E, Maring B, Kutner SE, Fulton RS, Lee MM, Ambrosone CB, Caan BJ (2009). Epidemiology of breast cancer subtypes in two prospective cohort studies of breast cancer survivors. Breast Cancer Res.

[9] Atchley DP, Albarracin CT, Lopez A, Valero V, Amos CI, Gonzalez-Angulo AM, Hortobagyi GN, Arun BK (2008). Clinical and pathologic characteristics of patients with BRCA-positive and BRCA-negative breast cancer. J Clin Oncol.

[10] Foulkes WD, Stefansson IM, Chappuis PO, Begin LR, Goffin JR, Wong N, Trudel M, Akslen LA (2003). Germline BRCA1 mutations and a basal epithelial phenotype in breast cancer. J Natl Cancer Inst.

[11] Comen E, Davids M, Kirchhoff T, Hudis C, Offit K, Robson M (2011). Relative contributions of BRCA1 and BRCA2 mutations to “triple-negative” breast cancer in Ashkenazi women. Breast Cancer Res Treat.

[12] Villarreal-Garza C, Weitzel JN, Llacuachaqui M, Sifuentes E, Magallanes-Hoyos MC, Gallardo L, Alvarez-Gomez RM, Herzog J, Castillo D, Royer R (2015). The prevalence of BRCA1 and BRCA2 mutations among young Mexican women with triple-negative breast cancer. Breast Cancer Res Treat.

[13] Greenup R, Buchanan A, Lorizio W, Rhoads K, Chan S, Leedom T, King R, McLennan J, Crawford B, Kelly Marcom P, Shelley Hwang E (2013). Prevalence of BRCA mutations among women with triple-negative breast cancer (TNBC) in a genetic counseling cohort. Ann Surg Oncol.

The article "Therapeutic landscape in mutational triple negative breast cancer" was published in 2018. Journal: Mol Cancer.

[14] Young SR, Pilarski RT, Donenberg T, Shapiro C, Hammond LS, Miller J, Brooks KA, Cohen S, Tenenholz B, DeSai D (2009). The prevalence of BRCA1 mutations among young women with triple-negative breast cancer. BMC Cancer.

[15] Cybulski C, Kluzniak W, Huzarski T, Wokolorczyk D, Kashyap A, Jakubowska A, Szwiec M, Byrski T, Debniak T, Gorski B (2015). Clinical outcomes in women with breast cancer and a PALB2 mutation: a prospective cohort analysis. Lancet Oncol.

[16] Heikkinen T, Karkkainen H, Aaltonen K, Milne RL, Heikkila P, Aittomaki K, Blomqvist C, Nevanlinna H (2009). The breast cancer susceptibility mutation PALB2 1592delT is associated with an aggressive tumor phenotype. Clin Cancer Res.

[17] Neidhardt G, Hauke J, Ramser J, Gross E, Gehrig A, Muller CR, Kahlert AK, Hackmann K, Honisch E, Niederacher D (2017). Association between loss-of-function mutations within the FANCM gene and Early-onset familial breast Cancer. JAMA Oncol.

[18] Kiiski JI, Pelttari LM, Khan S, Freysteinsdottir ES, Reynisdottir I, Hart SN, Shimelis H, Vilske S, Kallioniemi A, Schleutker J (2014). Exome sequencing identifies FANCM as a susceptibility gene for triple-negative breast cancer. Proc Natl Acad Sci U S A.

[19] Sun J, Meng H, Yao L, Lv M, Bai J, Zhang J, Wang L, Ouyang T, Li J, Wang T (2017). Germline mutations in cancer susceptibility genes in a large series of unselected breast cancer patients. Clin Cancer Res.

[20] Cancer Genome Atlas Network. Comprehensive molecular portraits of human breast tumours. Nature. 2012;490:61–70.10.1038/nature11412PMC346553223000897

[21] Santarpia L, Qi Y, Stemke-Hale K, Wang B, Young EJ, Booser DJ, Holmes FA, O'Shaughnessy J, Hellerstedt B, Pippen J (2012). Mutation profiling identifies numerous rare drug targets and distinct mutation patterns in different clinical subtypes of breast cancers. Breast Cancer Res Treat.

[22] Herschkowitz JI, He X, Fan C, Perou CM (2008). The functional loss of the retinoblastoma tumour suppressor is a common event in basal-like and luminal B breast carcinomas. Breast Cancer Res.

[23] Jones RA, Robinson TJ, Liu JC, Shrestha M, Voisin V, Ju Y, Chung PED, Pellecchia G, Fell VL, Bae S (2016). RB1 deficiency in triple-negative breast cancer induces mitochondrial protein translation. J Clin Invest.

[24] Shah SP, Roth A, Goya R, Oloumi A, Ha G, Zhao Y, Turashvili G, Ding J, Tse K, Haffari G (2012). The clonal and mutational evolution spectrum of primary triple-negative breast cancers. Nature.

[25] Dey N, De P, Leyland-Jones B (2017). PI3K-AKT-mTOR inhibitors in breast cancers: from tumor cell signaling to clinical trials. Pharmacol Ther.

The article "Therapeutic landscape in mutational triple negative breast cancer" was published in 2018. Journal: Mol Cancer.

[26] Xu H, Eirew P, Mullaly SC, Aparicio S (2014). The omics of triple-negative breast cancers. Clin Chem.

[27] Weisman PS, Ng CK, Brogi E, Eisenberg RE, Won HH, Piscuoglio S, De Filippo MR, Ioris R, Akram M, Norton L (2016). Genetic alterations of triple negative breast cancer by targeted next-generation sequencing and correlation with tumor morphology. Mod Pathol.

[28] Marotti JD, de Abreu FB, Wells WA, Tsongalis GJ (2017). Triple-negative breast cancer: next-generation sequencing for target identification. Am J Pathol.

[29] Stephens PJ, Tarpey PS, Davies H, Van Loo P, Greenman C, Wedge DC, Nik-Zainal S, Martin S, Varela I, Bignell GR (2012). The landscape of cancer genes and mutational processes in breast cancer. Nature.

[30] Nik-Zainal S, Davies H, Staaf J, Ramakrishna M, Glodzik D, Zou X, Martincorena I, Alexandrov LB, Martin S, Wedge DC (2016). Landscape of somatic mutations in 560 breast cancer whole-genome sequences. Nature.

[31] Banerji S, Cibulskis K, Rangel-Escareno C, Brown KK, Carter SL, Frederick AM, Lawrence MS, Sivachenko AY, Sougnez C, Zou L (2012). Sequence analysis of mutations and translocations across breast cancer subtypes. Nature.

[32] Humphreys RC, Hennighausen L (2000). Transforming growth factor alpha and mouse models of human breast cancer. Oncogene.

[33] Kawazu M, Kojima S, Ueno T, Totoki Y, Nakamura H, Kunita A, Qu W, Yoshimura J, Soda M, Yasuda T (2017). Integrative analysis of genomic alterations in triple-negative breast cancer in association with homologous recombination deficiency. PLoS Genet.

[34] Morganella S, Alexandrov LB, Glodzik D, Zou X, Davies H, Staaf J, Sieuwerts AM, Brinkman AB, Martin S, Ramakrishna M (2016). The topography of mutational processes in breast cancer genomes. Nat Commun.

[35] Hartmaier RJ, Priedigkeit N, Lee AV (2012). Who’s driving anyway? Herculean efforts to identify the drivers of breast cancer. Breast Cancer Res.

[36] Kobayashi K, Ito Y, Matsuura M, Fukada I, Horii R, Takahashi S, Akiyama F, Iwase T, Hozumi Y, Yasuda Y, Hatake K (2016). Impact of immunohistological subtypes on the long-term prognosis of patients with metastatic breast cancer. Surg Today.

[37] Yam C, Mani SA, Moulder SL (2017). Targeting the molecular subtypes of triple negative breast cancer: understanding the diversity to progress the field. Oncologist.

[38] Kim C, Gao R, Sei E, Brandt R, Hartman J, Hatschek T, Crosetto N, Foukakis T, Navin NE (2018). Chemoresistance evolution in triple-negative breast cancer delineated by single-cell sequencing. Cell.

[39] von Minckwitz G, Schneeweiss A, Loibl S, Salat C, Denkert C, Rezai M, Blohmer JU, Jackisch C, Paepke S, Gerber B (2014). Neoadjuvant carboplatin in patients with triple-negative and HER2-positive early breast cancer (GeparSixto; GBG 66): a randomised phase 2 trial. Lancet Oncol.

The article "Therapeutic landscape in mutational triple negative breast cancer" was published in 2018. Journal: Mol Cancer.

[40] Sikov WM, Berry DA, Perou CM, Singh B, Cirrincione CT, Tolaney SM, Kuzma CS, Pluard TJ, Somlo G, Port ER (2015). Impact of the addition of carboplatin and/or bevacizumab to neoadjuvant once-per-week paclitaxel followed by dose-dense doxorubicin and cyclophosphamide on pathologic complete response rates in stage II to III triple-negative breast cancer: CALGB 40603 (alliance). J Clin Oncol.

[41] Minckwitz GV, Loibl S, Schneeweiss A, Salat CT, Rezai M, Zahm DM, Klare P, Blohmer JU, Tesch H, Khandan F (2016). Abstract S2–04: early survival analysis of the randomized phase II trial investigating the addition of carboplatin to neoadjuvant therapy for triple-negative and HER2-positive early breast cancer (GeparSixto). Cancer Res.

[42] Sikov WM, Berry DA, Perou CM, Singh B, Cirrincione CT, Tolaney SM, Somlo G, Port ER, Qamar R, Sturtz K (2016). Abstract S2-05: event-free and overall survival following neoadjuvant weekly paclitaxel and dose-dense AC +/− carboplatin and/or bevacizumab in triple-negative breast cancer: outcomes from CALGB 40603 (alliance). Cancer Res.

[43] Tutt A, Ellis P, Kilburn L, Gilett C, Pinder S, Abraham J, Barrett S, Barrett-Lee P, Chan S, Cheang M (2015). Abstract S3–01: the TNT trial: a randomized phase III trial of carboplatin (C) compared with docetaxel (D) for patients with metastatic or recurrent locally advanced triple negative or <em>BRCA1/2</em> breast cancer (CRUK/07/012). Cancer Res.

[44] Tutt A, Robson M, Garber JE, Domchek SM, Audeh MW, Weitzel JN, Friedlander M, Arun B, Loman N, Schmutzler RK (2010). Oral poly(ADP-ribose) polymerase inhibitor olaparib in patients with BRCA1 or BRCA2 mutations and advanced breast cancer: a proof-of-concept trial. Lancet.

[45] Robson M, Im SA, Senkus E, Xu B, Domchek SM, Masuda N, Delaloge S, Li W, Tung N, Armstrong A (2017). Olaparib for metastatic breast Cancer in patients with a germline BRCA mutation. N Engl J Med.

[46] Rugo HS, Olopade OI, DeMichele A, Yau C, van’t Veer LJ, Buxton MB, Hogarth M, Hylton NM, Paoloni M, Perlmutter J (2016). Adaptive randomization of veliparib-carboplatin treatment in breast cancer. N Engl J Med.

[47] Gadhikar MA, Sciuto MR, Alves MV, Pickering CR, Osman AA, Neskey DM, Zhao M, Fitzgerald AL, Myers JN, Frederick MJ (2013). Chk1/2 inhibition overcomes the cisplatin resistance of head and neck cancer cells secondary to the loss of functional p53. Mol Cancer Ther.

[48] Wang Q, Fan S, Eastman A, Worland PJ, Sausville EA, O'Connor PM (1996). UCN-01: a potent Abrogator of G 2 checkpoint function in Cancer cells with disrupted p53. JNCI.

The article "Therapeutic landscape in mutational triple negative breast cancer" was published in 2018. Journal: Mol Cancer.

[49] Bouwman P, Jonkers J (2012). The effects of deregulated DNA damage signalling on cancer chemotherapy response and resistance. Nat Rev Cancer.

[50] Ma CX, Cai S, Li S, Ryan CE, Guo Z, Schaiff WT, Lin L, Hoog J, Goiffon RJ, Prat A (2012). Targeting Chk1 in p53-deficient triple-negative breast cancer is therapeutically beneficial in human-in-mouse tumor models. J Clin Invest.

[51] Fracasso PM, Williams KJ, Chen RC, Picus J, Ma CX, Ellis MJ, Tan BR, Pluard TJ, Adkins DR, Naughton MJ (2011). A phase 1 study of UCN-01 in combination with irinotecan in patients with resistant solid tumor malignancies. Cancer Chemother Pharmacol.

[52] Hong D, Infante J, Janku F, Jones S, Nguyen LM, Burris H, Naing A, Bauer TM, Piha-Paul S, Johnson FM (2016). Phase I study of LY2606368, a checkpoint kinase 1 inhibitor, in patients with advanced Cancer. J Clin Oncol.

[53] Ma CX, Ellis MJ, Petroni GR, Guo Z, Cai SR, Ryan CE, Craig Lockhart A, Naughton MJ, Pluard TJ, Brenin CM (2013). A phase II study of UCN-01 in combination with irinotecan in patients with metastatic triple negative breast cancer. Breast Cancer Res Treat.

[54] Ellis MJ, Perou CM (2013). The genomic landscape of breast Cancer as a therapeutic roadmap. Cancer Discov.

[55] Kumar A, Fernandez-Capetillo O, Carrera AC (2010). Nuclear phosphoinositide 3-kinase beta controls double-strand break DNA repair. Proc Natl Acad Sci U S A.

[56] Ibrahim YH, Garcia-Garcia C, Serra V, He L, Torres-Lockhart K, Prat A, Anton P, Cozar P, Guzman M, Grueso J (2012). PI3K inhibition impairs BRCA1/2 expression and sensitizes BRCA-proficient triple-negative breast cancer to PARP inhibition. Cancer Discov.

[57] Andre F, O'Regan R, Ozguroglu M, Toi M, Xu B, Jerusalem G, Masuda N, Wilks S, Arena F, Isaacs C (2014). Everolimus for women with trastuzumab-resistant, HER2-positive, advanced breast cancer (BOLERO-3): a randomised, double-blind, placebo-controlled phase 3 trial. Lancet Oncol.

[58] Hurvitz SA, Andre F, Jiang Z, Shao Z, Mano MS, Neciosup SP, Tseng LM, Zhang Q, Shen K, Liu D (2015). Combination of everolimus with trastuzumab plus paclitaxel as first-line treatment for patients with HER2-positive advanced breast cancer (BOLERO-1): a phase 3, randomised, double-blind, multicentre trial. Lancet Oncol.

[59] Wong SW, Tiong KH, Kong WY, Yue YC, Chua CH, Lim JY, Lee CY, Quah SI, Fow C, Chung C (2011). Rapamycin synergizes cisplatin sensitivity in basal-like breast cancer cells through up-regulation of p73. Breast Cancer Res Treat.

[60] De P, Sun Y, Carlson JH, Friedman LS, Leyland-Jones BR, Dey N (2014). Doubling down on the PI3K-AKT-mTOR pathway enhances the antitumor efficacy of PARP inhibitor in triple negative breast cancer model beyond BRCA-ness. Neoplasia.

The article "Therapeutic landscape in mutational triple negative breast cancer" was published in 2018. Journal: Mol Cancer.

[61] Gonzalez-Angulo AM, Akcakanat A, Liu S, Green MC, Murray JL, Chen H, Palla SL, Koenig KB, Brewster AM, Valero V (2014). Open-label randomized clinical trial of standard neoadjuvant chemotherapy with paclitaxel followed by FEC versus the combination of paclitaxel and everolimus followed by FEC in women with triple receptor-negative breast cancerdagger. Ann Oncol.

[62] Basho RK, Gilcrease M, Murthy RK, Helgason T, Karp DD, Meric-Bernstam F, Hess KR, Herbrich SM, Valero V, Albarracin C (2017). Targeting the PI3K/AKT/mTOR pathway for the treatment of mesenchymal triple-negative breast Cancer: evidence from a phase 1 trial of mTOR inhibition in combination with liposomal doxorubicin and bevacizumab. JAMA Oncol.

[63] Schuler M, Awada A, Harter P, Canon JL, Possinger K, Schmidt M, De Greve J, Neven P, Dirix L, Jonat W (2012). A phase II trial to assess efficacy and safety of afatinib in extensively pretreated patients with HER2-negative metastatic breast cancer. Breast Cancer Res Treat.

[64] Finn RS, Press MF, Dering J, Arbushites M, Koehler M, Oliva C, Williams LS, Di Leo A (2009). Estrogen receptor, progesterone receptor, human epidermal growth factor receptor 2 (HER2), and epidermal growth factor receptor expression and benefit from lapatinib in a randomized trial of paclitaxel with lapatinib or placebo as first-line treatment in HER2-negative or unknown metastatic breast cancer. J Clin Oncol.

[65] Tilch E, Seidens T, Cocciardi S, Reid LE, Byrne D, Simpson PT, Vargas AC, Cummings MC, Fox SB, Lakhani SR, Chenevix Trench G (2014). Mutations in EGFR, BRAF and RAS are rare in triple-negative and basal-like breast cancers from Caucasian women. Breast Cancer Res Treat.

[66] Jacot W, Lopez-Crapez E, Thezenas S, Senal R, Fina F, Bibeau F, Romieu G, Lamy PJ (2011). Lack of EGFR-activating mutations in European patients with triple-negative breast cancer could emphasise geographic and ethnic variations in breast cancer mutation profiles. Breast Cancer Res.

[67] Teng YH, Tan WJ, Thike AA, Cheok PY, Tse GM, Wong NS, Yip GW, Bay BH, Tan PH (2011). Mutations in the epidermal growth factor receptor (EGFR) gene in triple negative breast cancer: possible implications for targeted therapy. Breast Cancer Res.

[68] Lv N, Lin S, Xie Z, Tang J, Ge Q, Wu M, Xie X, Xie X, Wei W (2012). Absence of evidence for epidermal growth factor receptor and human homolog of the Kirsten rat sarcoma-2 virus oncogene mutations in breast cancer. Cancer Epidemiol.

[69] Toyama T, Yamashita H, Kondo N, Okuda K, Takahashi S, Sasaki H, Sugiura H, Iwase H, Fujii Y (2008). Frequently increased epidermal growth factor receptor (EGFR) copy numbers and decreased BRCA1 mRNA expression in Japanese triple-negative breast cancers. BMC Cancer.

The article "Therapeutic landscape in mutational triple negative breast cancer" was published in 2018. Journal: Mol Cancer.

[70] Cao WM, Gao Y, Wang XJ (2015). Lack of epidermal growth factor receptor (EGFR)-activating mutations in triple-negative breast cancer in China. Breast Cancer Res.

[71] Johnson J, Thijssen B, McDermott U, Garnett M, Wessels LF, Bernards R (2016). Targeting the RB-E2F pathway in breast cancer. Oncogene.

[72] Kaelin WG (2003). E2F1 as a target: promoter-driven suicide and small molecule modulators. Cancer Biol Ther.

[73] Duncan JS, Whittle MC, Nakamura K, Abell AN, Midland AA, Zawistowski JS, Johnson NL, Granger DA, Jordan NV, Darr DB, et al. Dynamic reprogramming of the kinome in response to targeted MEK inhibition in triple-negative breast cancer. Cell. 2012;149:307–21.10.1016/j.cell.2012.02.053PMC332878722500798

[74] Sabova L, Kretova M, Luciakova K (2013). New insights into the role of NF1 in cancer. Neoplasma.

[75] Balko JM, Schwarz LJ, Bhola NE, Kurupi R, Owens P, Miller TW, Gomez H, Cook RS, Arteaga CL (2013). Activation of MAPK pathways due to DUSP4 loss promotes cancer stem cell-like phenotypes in basal-like breast cancer. Cancer Res.

[76] Hoeflich KP, O'Brien C, Boyd Z, Cavet G, Guerrero S, Jung K, Januario T, Savage H, Punnoose E, Truong T (2009). In vivo antitumor activity of MEK and phosphatidylinositol 3-kinase inhibitors in basal-like breast cancer models. Clin Cancer Res.

[77] Mirzoeva OK, Das D, Heiser LM, Bhattacharya S, Siwak D, Gendelman R, Bayani N, Wang NJ, Neve RM, Guan Y (2009). Basal subtype and MAPK/ERK kinase (MEK)-phosphoinositide 3-kinase feedback signaling determine susceptibility of breast cancer cells to MEK inhibition. Cancer Res.

[78] Gonzalez-Angulo AM, Timms KM, Liu S, Chen H, Litton JK, Potter J, Lanchbury JS, Stemke-Hale K, Hennessy BT, Arun BK (2011). Incidence and outcome of <em>BRCA</em> mutations in unselected patients with triple receptor-negative breast Cancer. Clin Cancer Res.

[79] Hartman AR, Kaldate RR, Sailer LM, Painter L, Grier CE, Endsley RR, Griffin M, Hamilton SA, Frye CA, Silberman MA (2012). Prevalence of BRCA mutations in an unselected population of triple-negative breast cancer. Cancer.

[80] Sharma P, Klemp JR, Kimler BF, Mahnken JD, Geier LJ, Khan QJ, Elia M, Connor CS, McGinness MK, Mammen JM (2014). Germline BRCA mutation evaluation in a prospective triple-negative breast cancer registry: implications for hereditary breast and/or ovarian cancer syndrome testing. Breast Cancer Res Treat.

[81] Tung N, Battelli C, Allen B, Kaldate R, Bhatnagar S, Bowles K, Timms K, Garber JE, Herold C, Ellisen L (2015). Frequency of mutations in individuals with breast cancer referred for BRCA1 and BRCA2 testing using next-generation sequencing with a 25-gene panel. Cancer.

The article "Therapeutic landscape in mutational triple negative breast cancer" was published in 2018. Journal: Mol Cancer.

[82] Wong-Brown MW, Meldrum CJ, Carpenter JE, Clarke CL, Narod SA, Jakubowska A, Rudnicka H, Lubinski J, Scott RJ (2015). Prevalence of BRCA1 and BRCA2 germline mutations in patients with triple-negative breast cancer. Breast Cancer Res Treat.

[83] Gonzalez-Rivera M, Lobo M, Lopez-Tarruella S, Jerez Y, Del Monte-Millan M, Massarrah T, Ramos-Medina R, Ocana I, Picornell A, Garzon SS (2016). Frequency of germline DNA genetic findings in an unselected prospective cohort of triple-negative breast cancer patients participating in a platinum-based neoadjuvant chemotherapy trial. Breast Cancer Res Treat.

[84] Zhang J, Sun J, Chen J, Yao L, Ouyang T, Li J, Wang T, Fan Z, Fan T, Lin B, Xie Y (2016). Comprehensive analysis of BRCA1 and BRCA2 germline mutations in a large cohort of 5931 Chinese women with breast cancer. Breast Cancer Res Treat.

[85] Yang XR, Devi BCR, Sung H, Guida J, Mucaki EJ, Xiao Y, Best A, Garland L, Xie Y, Hu N (2017). Prevalence and spectrum of germline rare variants in BRCA1/2 and PALB2 among breast cancer cases in Sarawak, Malaysia. Breast Cancer Res Treat.

[86] Wong-Brown MW, Avery-Kiejda KA, Bowden NA, Scott RJ (2014). Low prevalence of germline PALB2 mutations in Australian triple-negative breast cancer. Int J Cancer.

[87] Ollier M, Radosevic-Robin N, Kwiatkowski F, Ponelle F, Viala S, Privat M, Uhrhammer N, Bernard-Gallon D, Penault-Llorca F, Bignon YJ, Bidet Y (2015). DNA repair genes implicated in triple negative familial non-BRCA1/2 breast cancer predisposition. Am J Cancer Res.

[88] Hahnen E, Lederer B, Hauke J, Loibl S, Krober S, Schneeweiss A, Denkert C, Fasching PA, Blohmer JU, Jackisch C (2017). Germline mutation status, pathological complete response, and disease-free survival in triple-negative breast Cancer: secondary analysis of the GeparSixto randomized clinical trial. JAMA Oncol.

